The article "Bovine Lactoferrin Induces Cell Death in Human Prostate Cancer Cells" was published in 2022. Journal: Oxid Med Cell Longev.

# Bovine Lactoferrin Induces Cell Death in Human Prostate Cancer Cells

**DOI:** 10.1155/2022/2187696

**Published:** 2022-09-02

**Authors:** Vanessa P. Rocha, Samir P. C. Campos, Caroline A. Barros, Pablo Trindade, Leticia R. Q. Souza, Triciana G. Silva, Etel R. P. Gimba, Anderson J. Teodoro, Rafael B. Gonçalves

**Affiliations:** ^1^Department of Biochemistry, Biomedical Institute, UNIRIO, 20211-040, Brazil; ^2^Cell and Molecular Biology Graduate Program, UNIRIO, 20211-040, Brazil; ^3^Medical Biochemistry Institute, UFRJ, 21941-590, Brazil; ^4^Multicentre Graduate Program in Biochemistry and Molecular Biology, IFRJ, 20270-021, Brazil; ^5^D'Or Institute for Research and Education-IDOR, 22281-100, Brazil; ^6^National Center for Structural Biology and Bioimaging, CENABIO, UFRJ, 21941-902, Brazil; ^7^Natural Science Department, UFF, 28895-532, Brazil; ^8^Cellular and Molecular Oncology Program, National Institute of Cancer (INCA), 20231-050, Brazil; ^9^Department of Nutrition and Dietetics, UFF, 22290-250, Brazil

## Abstract

Bovine lactoferrin (bLf) is a multifunctional protein widely associated with anticancer activity. Prostate cancer is the second most frequent type of cancer worldwide. This study was aimed at evaluating the influence of bLf on cell viability, cell cycle progression, reactive oxygen species (ROS) production, and rate of apoptosis in the human prostate cancer cell line (DU-145). MTT assay and trypan blue exclusion were used to analyze cell viability. Morphological changes were analyzed through optical microscopy after 24 h and 48 h of bLf treatment. FITC-bLf internalization and cellular damage were observed within 24 h by confocal fluorescence microscopy. Cell cycle analyses were performed by flow cytometry and propidium iodide. For caspases 3/7 activation and reactive oxygen species production evaluation, cells were live-imaged using the high-throughput system Operetta. The cell viability assays demonstrated that bLf induces cell death and morphological changes after 24 h and 48 h of treatment compared to control on DU-145 cells. The bLf internalization was detected in DU-145 cells, G_1_-phase arrest of the cell cycle, caspase 3/7 activation, and increased oxidative stress on bLf-treated cells. Our data support that bLf has an important anticancer activity, thus offering new perspectives in preventing and treating prostate cancer.

## 1. Introduction

Bovine Lactoferrin (bLf) is found in cattle and is an iron-bounding protein. bLf is present in several exocrine secretions, such as tears, saliva, milk, and cervical mucus. It has a molecular mass of approximately 80 kDa [1, 2]. This protein can be found in two conformational states. The conformational state “apo-” (apo-bLf) represents the protein not bound to ferric ions, while the conformational state “holo-” (holo-bLf) represents the protein bound to two ferric ions. Lf binds to the ferric ion in a very high affinity, approximately 10^−20^ M of affinity constant (*K_D_*), and some of its physiological functions rely on that iron-binding property. Holo-bLf has a more compact, stable structure and is less sensitive to thermal denaturation and proteolysis due to the iron bond in its structure, compared to apo-bLf [3–5]. bLf has proven to be a great model for studying biological activities, including iron transport, immunomodulatory, anti-inflammatory, antiviral, antioxidant, and antitumor properties. Due to its multiple biological functions, bLf structural changes have been widely associated with immune enhancement and anticarcinogenic properties [1, 4–6].

The article "Bovine Lactoferrin Induces Cell Death in Human Prostate Cancer Cells" was published in 2022. Journal: Oxid Med Cell Longev.

Currently, great attention has been given initiatives aimed at preventing cancer. This disease alone is the second leading cause of death in the United States and a major public health problem worldwide. Counting about 19.3 million new cases of cancer per year worldwide accounting for nearly 10 million deaths in 2020. The coronavirus disease 2019 (COVID-19) pandemic drastically affected the diagnosis and treatment of cancer, which has led to an increase in mortality rates [7–9].

Robust evidence points out bLf as a promising biomolecule in cancer research. For instance, a previous study reported that treatment with bLf could suppress colon carcinogenesis by inducing elevated Fas expression, activation of caspases 3 and 8, and inductance ion of DNA fragmentation, which led to apoptosis of cancer cells in rat colon mucosa [10, 11]. Similarly, other studies demonstrated that bLf decreased the growth of colon, lung, bladder, and breast cancer cells. Induction of apoptosis in colon, lung, stomach, and breast cancer cells has also been reported [11–19].

Prostate cancer is the leading cancer diagnosis among men and the third most common diagnosis overall, with 1,414,259 expected cases in 2020, the fifth leading cause of cancer death in the United States [7, 20].

Recent evidence reported that bLf inhibits proliferation, induces apoptosis and intracellular acidification, and disturbs lysosomal acidification in the PC-3 prostate cancer cell line. This work suggests that the bLf mechanism of action is mediated by the V-ATPase pump in the plasma membrane, hindering its activity and decreasing acidity, thus limiting prostate cancer progression and metastasis formation [21].

New treatment options for prostate cancer are being used, and several recent studies for its treatment are being conducted. However, despite all the advances, the morbidity and mortality of prostate cancer have increased worldwide [22]. Bioactive compounds have been associated with modifying specific carcinogenic processes [23]. Therefore, this study is aimed at evaluating the cytotoxic effects of bLf on its apo- and holo- forms in the DU-145 cell line of prostate cancer.

The article "Bovine Lactoferrin Induces Cell Death in Human Prostate Cancer Cells" was published in 2022. Journal: Oxid Med Cell Longev.

## 2. Materials and Methods

### 2.1. Standards and Chemicals

All chemicals used in this work were of analytical grade. The water was distilled and deionized using a Millipore water purification system. Bovine lactoferrin was purchased from Life Extension (Florida, USA). The nitrilotriacetic acid, ferric nitrate, and Dulbecco's cell culture medium was obtained from Sigma-Aldrich Chemical Company (St. Louis, MO). Fetal bovine serum was purchased from Gibco™, Thermo Fisher Scientific (Waltham, Massachusetts, EUA). Tissue culture flasks were purchased from Greiner Bio-One International GmbH (Kremsmünster, Austria).

### 2.2. Preparation of bLf Forms: Apo-Lactoferrin

Bovine apo-lactoferrin was prepared from capsules containing 300 mg of protein (Life Extension, USA). Phosphate saline buffer (PBS) (140 mM NaCl, 2.7 mM KCl, 10 mM Na_2_HPO_4_, and 1.8 mM KH_2_PO_4_ at pH 7.4) was used for protein solubilization. The capsule contained cellulose, and to separate it from the protein, four cycles of centrifugation of 10 minutes each was performed at an angular speed of 7000 rpm (12,052 × *g*) at 4°C. Then, apo-bLf was filtered using a sterile nitrocellulose membrane of a 0.22 *μ*m pore (Millipore, USA) in an ESCO biosafety cabin, aliquoted, and frozen at -20°C. Finally, apo-bLf concentration was measured by an absorbance spectrophotometer at a 280 nm wavelength, using a molar extinction coefficient of 1.27 [24, 25].

### 2.3. Preparation of bLf Forms: Holo-Lactoferrin

Holo-lactoferrin was prepared from apo-bLf [3]. Apo-bLf stock was diluted in 10 mM Tris buffer, 75 mM NaCl, and pH 7.2. After dilution, a FeNTA solution (9.9 mM ferric nitrate and 8.5 mM nitrilotriacetic acid, deionized water) was added in a 2 : 1 ratio (FeNTA:bLf solution). The pH of the solution was adjusted to 7.0 and incubated for one hour at 4°C. Subsequently, the sample was dialyzed against a buffer with 25 mM Tris, 150 mM NaCl pH 7.5 at 4°C for 48 h. A dialysis membrane with a cut-off of 10 kDa was used, and the buffer was changed every 5 h. Then, the holo-bLf was filtered on a sterile nitrocellulose membrane of a 0.22 *μ*m pore (Millipore, USA) in an ESCO biosafety cabin, aliquoted, and frozen at -20°C. Finally, the protein concentration was then measured in a spectrophotometer at a 280 nm wavelength, using the molar extinction coefficient of 1.51 holo-bLf. The presence of iron ions was verified using a spectrophotometric absorbance reading at 465 nm [3, 26, 27].

The article "Bovine Lactoferrin Induces Cell Death in Human Prostate Cancer Cells" was published in 2022. Journal: Oxid Med Cell Longev.

### 2.4. Cell Culture

The cell line was obtained from the Neoplastic Biomarkers Group (Nacional Institute of Cancer-INCA), which certified its identity and quality. The human prostate carcinoma cell line DU-145 (ATCC-HTB-81) was maintained routinely in high-glucose Dulbecco's Modified Eagle Medium (DMEM) (Sigma, New York, NY, USA), supplemented with a 10% fetal bovine serum (FBS) and 1% penicillin-streptomycin (PS) (Sigma, New York, NY, USA), pH 7.4, under 5% CO_2_ atmosphere and 37°C. Once the cells reached 80% of confluence, they were dissociated with a 0.05% trypsin-ethylenediamine tetraacetic acid (EDTA) and subcultured in 25 or 75 cm^2^ plastic flasks at a 25 × 10^4^ cells/cm^2^ density, every two days, following ATCC instructions.

### 2.5. Cell Viability Assays: MTT Assay

Cell viability was determined by a 3-(4,5-dimethylthiazol-2-yl)-2,5-diphenyltetrazolium bromide (MTT) colorimetric test (Amresco, USA) [28]. By this test, the quantification of MTT reduction in formazan characterizes a detection of metabolic activity that is linked to cell viability. 96-well plates were prepared using 1.0 × 10^4^ cells/well for this analysis. After 24 h, the cells were washed, and 100 *μ*L of apo- and holo-bLf solution was added to the wells at concentrations of 2, 4, 8, and 16 mg/mL (diluted in the culture medium described above). As a negative control, DMEM was used. After 24 h and 48 h of incubation, the bLf was removed, the wells were washed, and a solution of 200 *μ*L MTT (Sigma) was added in PBS. The plate was incubated for 3 hours at 37°C. After this period, the plate was analyzed on a spectrophotometer using absorbance at 570 nm and 650 nm. Wells with negative control were considered 100% in cell viability. Triton X-100 0.1% was used as a 100% death control to normalize calculations. This experiment was repeated in triplicate with independent preparations.

### 2.6. Cell Viability Assays: Cell Counting with Neubauer Chamber

The experiment is based on viable cells' selective permeability and was not stained by trypan blue since dead cells undergo changes in the membrane that affect their selective permeability, thus allowing the blue dye to enter [29]. The tests were performed by cultivating the cells in 24-well plates and kept with a 500 *μ*L of culture medium at 37°C until reaching a 90% confluence. Then, the medium was removed, and the cells were washed with PBS. The culture medium was placed in the control, and concentrations of apo-bLf and holo-bLf 2, 4, 8, and 16 mg/mL prepared with the culture medium were placed in their respective wells. After treatment for 24 h and 48 h, the cells were trypsinized and resuspended in a 200 *μ*L of the medium. 10 *μ*L of that suspension was collected and mixed with a 10 *μ*L of 0,4% trypan blue (Gibco) solution in PBS. 10 *μ*L was collected and placed in the Neubauer chamber for cell counting from the last suspension. Cells in the four outer quadrants were counted. Live and dead cells were distinguished by staining. Finally, cell concentration was calculated, and a percentage graph was made.

The article "Bovine Lactoferrin Induces Cell Death in Human Prostate Cancer Cells" was published in 2022. Journal: Oxid Med Cell Longev.

### 2.7. Cell Morphology Analysis

The analysis of cell morphology was carried out using images of cells in culture after 24 h and 48 h of treatment using both forms of bLf. The cells were placed in a 24-well plate. After reaching a 90% confluence, the culture medium was removed, and the cells were washed with warm PBS and incubated with concentrations of 0, 2, 4, 8, and 16 mg/mL apo- and holo-bLf for 24 h and 48 h. Images were obtained using an EVOS™ optical microscope (Thermo Fisher) and EVOSTM 20X Objective lens (PlanFluor INF/1.2). Three images per well were obtained, as to know: center, upper right quadrant, and lower left quadrant (close to the board's limit). Experiments were carried out in triplicate. Images were acquired at an image resolution of 1280 × 960 pixels, 24-bit RGB. By using Image J software (1.53c), images were first converted to an 8-bit monochrome image. Then, levels were adjusted to visualize the cell structures better, regulating the brightness and contrast curve. Images were calibrated to adapt to the actual pixel size using the Evos reference bar. Next, the bars were included, and the images were analyzed.

### 2.8. Bovine Lactoferrin Cell Internalization Assays

We performed the bLf labeling with fluorescein isothiocyanate (FITC) for cell internalization assays at a 1 : 10 molar ratio for one hour at 4°C. For the labeling process, lactoferrin was incubated in primary phosphate buffer (2.5% Na_2_HPO_4_.x7H_2_O and 0.082% NaH_2_PO_4_) at pH 8. To remove all free FITC, successive centrifugations using PBS at pH 7.4 (5 times) were performed using a Vivaspin filter unit (GE Health Care, USA) with a cut-off molecular weight of 30 kDa [30]. We proceeded with a sterile filtration of the labeled apo- and holo-bLf using a 0.22 *μ*m syringe-driven filter unit. The proteins were used on the same day for the experiments. The cells were plated on a commercial “CELLview™ Slide” plate (Greiner Bio-One) to proceed with the investigations. After an 80% confluence, the cells were washed with 100 *μ*L of PBS and incubated with apo- and holo-bLf-FITC conjugates (8 and 16 mg/mL) diluted in DMEM 4°C for 15 min. Subsequently, to remove unbound bLf, cells were washed with ice-cold PBS and immediately incubated with DMEM. After interaction with bLf, cells were kept under a 5% CO_2_ atmosphere and 37°C for 24 h. After treatment, the cells were washed with warm PBS and fixed with 3.7% paraformaldehyde in PBS for 15 minutes at room temperature. The study of lactoferrin cellular localization occurred through Laser Scanning Confocal Fluorescence Microscopy (LSCFM) using the LSM 510 Meta Confocal Microscope (Zeiss Inc., Oberkochen) and EC Plan-Neofluar 40x/1.30 Oil DIC M27 (Zeiss Inc.) objective lens.

The article "Bovine Lactoferrin Induces Cell Death in Human Prostate Cancer Cells" was published in 2022. Journal: Oxid Med Cell Longev.

### 2.9. Cell Cycle Analysis

Cell cycle analysis was performed using propidium iodide staining. The cells were plated on a 6-well plate, and after reaching a 90% confluence, cells were treated with 1.5 mL of apo-bLf and holo-bLf at concentrations of 2, 4, 8, and 16 mg/mL. Control cells were kept with a culture medium only. After 24 h and 48 h of bLf treatment, cells were washed with PBS and dissociated using trypsin. 1 × 10^5^ cells were collected from each treatment and mixed with cold Vindelov's solution [31]. After incubation for 15 minutes, protected from light, cell suspensions were analyzed using a BD FACSAria II cytometer (BD Biosciences). Twenty thousand events were then analyzed by flow cytometer on the fluorochrome PI channel (488 nm excitation laser and long pass filter 556 and band pass filter 616/23 for emission). Data were analyzed using the FlowJo™ v10.7.2 Software (BD Biosciences).

### 2.10. Analysis of Oxidative Stress and Activation of Apoptosis

The probe test for the assessment of oxidative stress and activation of apoptosis was carried out using the Operetta High-Content Imaging System and two different probe solutions, one containing the dihydroethidium (DHE) reagent (Thermo Fisher #D1168) and Hoechst 33342 (Thermo Fisher #H1399), with a final concentration of 5 *μ*M and 1 *μ*M, respectively. The other solution contained the reagent CellEvent™ Caspase-3/7 Green Detection Reagent (Thermo Fisher #C10423) and Hoechst 33342 (Thermo Fisher #H1399), with a final concentration of 2 *μ*M and 1 *μ*M. The cells were placed in a 96-well plate (Greiner Bio-One #655090). Each well had 2000 to 2500 cells. After 24 h of cell growth, the plates were treated with 100 *μ*L of apo-bLf and holo-bLf in 2, 4, 8, and 16 mg/mL for 24 h and 48 h. Then, the medium containing the compounds was removed. 50 *μ*L of the probe solutions was added with each solution in each specific plate, diluted with DMEM culture medium without phenol red. The plates were incubated at 37°C, 5% CO_2_ for 30 min, and placed in the Operetta High Content Imaging System (Perkin Elmer) at 37°C and a 5% CO_2_. The images were obtained with the 20x objective and high numerical openings (NA) (PerkinElmer, USA). Data were analyzed using the Harmony 5.1 high-content image analysis software (PerkinElmer, USA). Nine independent fields were evaluated from wells in triplicate by experimental conditions. The results were demonstrated with a bar graph showing the positive cells for caspase 3/7 and DHE.

The article "Bovine Lactoferrin Induces Cell Death in Human Prostate Cancer Cells" was published in 2022. Journal: Oxid Med Cell Longev.

### 2.11. Statistical Analysis

The results are presented as mean with the corresponding standard deviation. Data were analyzed using the statistical software GraphPad Prism (version 6.01, GraphPad Software, San Diego, CA). One-way variance (ANOVA) using the Bonferroni post hoc test at a confidence level of 95% was used to test cell viability, cell cycle, and apoptosis.

### 2.12. Graphical Scheme

Figure 1 shows the graphical scheme of the study approach. It contains all the methodologies used.

## 3. Results

### 3.1. bLf Induces Cell Death in the DU-145 Cell Line

The effect of both forms of bLf (apo-bLf and holo-bLf) on cell viability was evaluated by two different approaches, MTT assay and trypan blue exclusion test (Figure 2). The screening of cytotoxic activity demonstrated that apo-bLf and holo-bLf reduced DU-145 cell viability using MTT assay. No differences were detected between the control group and cells exposed to 2, 4, and 8 mg/mL apo-bLf following a 24 h treatment. However, we observed a decrease of 80% in average viability after a 48 h of apo-bLf exposure with 2 and 4 mg/mL and a reduction of 70% following an 8 mg/mL treatment. In addition, the highest concentration of apo-bLf (16 mg/mL) induced the most significant reduction in cell viability, up to 60% (*p* < 0.0001) and 40% (*p* < 0.01) after 24 h and 48 h, respectively (Figure 2(a)).

After 24 h, treatment with 2 and 4 mg/mL holo-bLf (Figure 2(b)) induced a reduction of 25% in cell viability compared to control (*p* < 0.05). After 48 h, no cytotoxic effects were observed following holo-bLf exposure (2 and 4 mg/mL). In contrast, the concentration of 8 mg/mL holo-bLf resulted in a drop in cell viability of 65% (*p* < 0.01) in 24 h and a decline of around 40% in 48 h (*p* < 0.05). Reductions of 50% and 90% of cell viability were observed using 16 mg/mL holo-bLf after 24 h and 48 h, respectively (*p* < 0.01).

To validate MTT findings, we also performed a trypan blue exclusion analysis to determine the number of viable cells in response to bLf treatment (Figures 2(c) and 2(d)). No significant difference in 24 h treatment with apo-bLf on all tested concentrations was observed (Figure 2(c)). However, after a 48 h treatment, we observed a reduction in cell viability of 30% (*p* < 0.01), 40% (*p* < 0.001), and more than 80% (*p* < 0.0001) following 4, 8, and 16 mg/mL apo-bLf, respectively. No significant differences were observed in lower concentrations of holo-bLf (2, 4, and 8 mg/mL) after 24 h treatment (Figure 2(d)). In turn, 16 mg/mL holo-bLf resulted in a 50% reduction in cell viability (*p* < 0.0001). Following 48 h treatment, a reduction in cell viability by approximately 40% (*p* < 0.001), 20% (*p* < 0.01), 60% (*p* < 0.0001), and 80% (*p* < 0.0001) was observed when using of 2, 4, 8, and 16 mg/mL holo-bLf, respectively.

The article "Bovine Lactoferrin Induces Cell Death in Human Prostate Cancer Cells" was published in 2022. Journal: Oxid Med Cell Longev.

### 3.2. bLf Causes Morphological Changes in the DU-145 Cell Line

In addition to the robust reduction in cell viability upon bLf treatment in the DU-145 cell line, evident changes in the morphology of the remaining cells (Figure 3) were observed. Treatment with both apo- and holo-bLf affected the cell shape so that most cells exhibited a stretched morphology and a reduced cell area (Figure 3(a)).

In addition, an increase in the number of intracellular granules could be primarily seen in the concentration of 16 mg/mL 24 h posttreatment and of 8 mg/mL 48 h posttreatment (Figure 3(b)). It is important to note that these morphological changes were more pronounced at 8 mg/mL with holo-bLf when compared to apo-bLf treatment.

### 3.3. bLf Internalizes and Causes DU-145 Cell Damage

Once we found that bLf induced DU-145 cell morphological changes and cell death, we then tested whether apo- and holo-bLf forms were internalized in DU-145 cells. For that, bLf forms were stained with FITC, and the images were obtained after 24 h of bLf treatment (Figure 4).

Using a fluorescence confocal microscope, we observed that FITC-stained apo- and holo-bLf were internalized at both tested concentrations. Moreover, lactoferrin internalization was more efficient in the highest concentration (16 mg/mL) of apo- and holo-bLf.

### 3.4. bLf Induces Cell Cycle Arrest in DU-145 Cells

We then aimed to evaluate whether the internalized apo- and holo-bLf were able to alter the cell cycle of DU-145 cells.  Table 1 demonstrates that treatment with 16 mg/mL of holo-bLf increased 22.9% and 29.4% the percentage of cells in the G_0_/G_1_ phase compared to control cells in 24 h and 48 h, respectively. The increase of cells in the G_0_/G_1_ phase was higher following a 48 h exposure than a 24 h. Apo-bLf treatment did not show any statistical difference in cell cycle distribution compared to control.

### 3.5. bLf Treatment Induces an Increase in Oxidative Stress and Activates Caspases 3/7 in the DU-145 Cell Line

We further investigated how bLf inhibited cell cycle progression and decreased cell viability.  Figure 5 is aimed at verifying possible oxidative stress changes and apoptosis activation induced by bLf in DU-145 cells. Live probes for reactive oxidative species (ROS) and apoptosis, DHE, and caspase 3/7 were used in a High-Content Imaging System to quantify these physiological changes.

The article "Bovine Lactoferrin Induces Cell Death in Human Prostate Cancer Cells" was published in 2022. Journal: Oxid Med Cell Longev.

Figures 5(a) and (b) show that both apo- and holo-bLf exposure increased DHE labelling when compared to the control. In 24 h, treatment with apo-bLf showed an increase of DHE-positive cells, being 7% with 2 mg/mL (*p* < 0.01), 12% with 4 mg/mL (*p* < 0.0001), 17% with 8 mg/mL (*p* < 0.0001), and 21% with 16 mg/mL (*p* < 0.0001) treatments. Holo-bLf also showed an increase of DHE-positive cells, being 8.5% with 2 mg/mL (*p* < 0.01), 11% with 4 mg/mL (*p* < 0.0001), 16% with 8 mg/mL (*p* < 0.0001), and 23% with 16 mg/mL (*p* < 0.0001) concentrations. After 48 h treatment, only holo-bLf with 16 mg/mL showed statistical difference in relation to control, increasing up to 12% the DHE-positive cells population.

In 24 h and 48 h treatments, we observed a concentration-dependent effect of both bLf forms on increasing DHE labeling. However, both apo- and holo-bLf structures exhibited higher increases in DHE labeling after 24 h in comparison to 48 h treatment.

On the other hand, the detection of activated caspases 3/7 was higher following a 48 h exposure with bLf than the 24 h experimental group (Figures 5(c) and 5(d)). After 24 h, apo-bLf showed an increase in activated caspases 3/7 labelling on concentrations of 8 mg/mL with 7.3% of positive cells (*p* < 0.001) and 16 mg/mL 10% (*p* < 0.0001) compared to the control group. At the same time of treatment, 24 h, holo-bLf induced caspase 3/7 activation only on the treatment using 16 mg/mL, thus presenting a 16.5% of activated caspase-positive cells.

After a 48 h of bLf treatment, apo-bLf demonstrated a dose-dependent caspase activation, showing the percentage of activated caspase 3/7 positive cells of 6.3% with 4 mg/mL (*p* < 0.01), 20.5% with 8 mg/mL (*p* < 0.0001), and 34% with 16 mg/mL (*p* < 0.0001). In addition, holo-bLf-treated cells also presented a dose dependent on caspase activation, with 10% with 4 mg/mL (*p* < 0.05), 28% with 8 mg/mL (*p* < 0.0001), and 49% with 16 mg/mL (*p* < 0.0001). At this stage, holo-bLf presented a higher effect on DU-145 caspases 3/7 activation than apo-bLf.

## 4. Discussion

Prostate cancer significantly challenges the health systems in many parts of the world. Even with a high survival rate when it is circumscribed, metastatic prostate cancer is primarily incurable even after discovering so many types of therapies. Despite all the efforts, prostate cancer is still one of the most frequent and lethal types of cancer. One of the most significant difficulties in reducing mortality is the lack of a broad spectrum of effective therapies against the considerable tumor heterogeneity at genetic and cellular levels, a considerable disease feature. Therefore, studies for the prevention and treatment of cancer are critical and have expanded over the years. There is still a demand for the development of compound effective for the induction of specific cell death [32, 33].

The article "Bovine Lactoferrin Induces Cell Death in Human Prostate Cancer Cells" was published in 2022. Journal: Oxid Med Cell Longev.

The structure of apo- and holo-bLf and differences in structural stability were investigated by our research group previously. This work showed that the presence of the iron ion in the holo-bLf structure promotes changes in its tertiary structure, when evaluating the tryptophan microenvironments and the interaction with the extrinsic fluorescent probe bis-ANS. In addition, holo-bLf has shown to have greater structural stability against chemical and physical disruptors [34].

Previous studies reported substantial antitumor effects of bLf, explicitly targeting tumor cells with no side effects on nontumorigenic cell lines (normal human intestinal epithelial cells and fibroblast). It has been shown that a semisaturated iron bLf (with 21% iron ions) is an important antitumor compound, as it selectively inhibits PC-3 cell growth at a concentration of 14 mg/mL. Based on this study, the concentrations used in this work were chosen better to achieve the desired antitumor bLf effect [21, 35].

Even though some studies demonstrated the antitumor bLf activity [17, 21, 35–37], little is known about the possible effects and differences of the two conformational states, holo- and apo-bLf. Therefore, we sought to compare them to better understand these differences in antitumor activity.

To investigate the cytotoxic effects of bLf, we performed an MTT assay and trypan blue exclusion. It was possible to observe that cell viability decreased in a dose- and time-dependent manner when compared to control, and these effects were more intense following holo-bLf exposure (Figure 2).

A previous study on antitumor activity was developed with conjugation of bLf and doxorubicin in prostate cancer cell lines. The conjugation of both molecules proved to be more effective against cancer development by increasing cytotoxicity to cancer cells but presenting lower toxicity to normal cells compared to doxorubicin-treated cells alone [32].

Morphological changes induced by bLf treatment were characterized by an increase in the number of intracellular granules and induction of stretched morphology (Figure 3). Few cells were left in bLf-treated wells to confirm the viability results. Together, these results demonstrate that bLf affects the cell morphology of DU-145 cells compared to the control. Although both apo- and holo-bLf cause similar morphological changes in dose- and time-dependent effects, treatment with holo-bLf showed to be more robust when compared to apo-bLf treatment.

The article "Bovine Lactoferrin Induces Cell Death in Human Prostate Cancer Cells" was published in 2022. Journal: Oxid Med Cell Longev.

The internalization of apo- and holo-bLf in the DU-145 cell line allowed us to infer that both bLf forms possibly interact with intracellular targets (Figure 4). This type of interaction between DU-145 cells and bLf can be explained because this protein has a positive charge in the N-terminal region that can interact with the negative charge of heparin and glycosaminoglycans present on cell surfaces [30, 38]. In addition, it is already known that lactoferrin can bind to low-density lipoprotein receptors and proteins related to the low-density lipoprotein receptor [38]. Another way of cellular bLf internalization that has been highly characterized is facilitated by receptor-mediated endocytosis, and then, bLf enters the endo-lysosome [32, 39, 40].

Cancer diseases characteristically induce alterations of normal growth signaling pathways. Tumor cells present a growth advantage since the regulators that govern the progression of the G_1_ phase of the cell cycle are natural oncogenesis targets. Therefore, analysis of the cell cycle progression has been pointed out as an essential tool for identifying new antitumor treatments. A decrease in cell division can inhibit tumor growth, thus inducing a delay in cancer development. Many studies that aim to propose antitumor remedies observed cell arrest in the G_0_/G_1_ phase and other results [41–43].

During the present work, we also quantified the percentage of cells at different cell cycle stages upon bLf administration (Table 1). In our culture conditions, most DU-145 cell lines showed to be at the G_0_/G_1_ phase, which accounts for ~45% of cells. The administration of apo-bLf does not modulate the DU-145 cell cycle on all concentrations and treatment times analyzed, although increasing G_0_/G_1_ population was observed upon a 16 mg/mL treatment. In turn, holo-bLf showed a dependent concentration increase in cells at G_0_/G_1_, which was even higher than the observed with apo-bLf exposure, which accounts for a ~75% of cells in a 16 mg/mL, thus showing that holo-bLf induces cell cycle arrest at the G_0_/G_1_ phase.

Previous studies showed that bLf induces cell cycle arrest at the G_0_/G_1_ phase in highly metastatic oral mucosa and breast cancer cells [44, 45]. Our preliminary results corroborate previous findings described in the literature concerning the action of bLf and suggest that this protein may affect the cell cycle of cancer cells.

Detection of oxidative stress was carried out using DHE, a fluorescent probe used to detect ROS, as it undergoes a nonspecific oxidation process [46]. Our results (Figure 5) showed that bLf treatment increased oxidative stress levels in DU-145 cells in 24 h. This could be related to oxidative stress-induced cancer cell death. These data are in accordance with other published data that also showed increased ROS levels in less than 24 h upon Lf treatment in cancer cell lines [47, 48]. However, unlike most published data, we decided to perform ROS production analysis up to 48 h post bLf treatment. Although there is a dose-dependent increase in ROS production after a 24 h of bLf treatment, ROS levels at 48 h are smaller than at 24 h. Those data suggest that the ROS production induced by bLf could be transitory and time-dependent.

The article "Bovine Lactoferrin Induces Cell Death in Human Prostate Cancer Cells" was published in 2022. Journal: Oxid Med Cell Longev.

This difference could be explained, at least partially, because of bLf availability. In this context, cells could consume bLf or degrade in medium at the initial, thus supporting ROS production at 24 h but not at 48 h. Moreover, due to the chronology of the events, ROS detected in 24 h may be the inducer of cell death observed in 48 h. Therefore, those affected by bLf died. In holo-bLf-treated cells, lower levels of ROS in 48 h than 24 h were detected but higher than apo-bLf at the same time. Unpublished results from our group showed that holo-bLf presented more excellent structural stability than apo-bLf, which could be why we can still see the effect of this protein even after 48 h of treatment.

ROS plays an important role in cancer and is usually associated with promoting protumorigenic signaling, thus facilitating cancer cell proliferation, survival, and adaptation to hypoxia. Nevertheless, ROS can also promote antitumorigenic signaling and trigger oxidative stress-induced cancer cell death. Compared with normal cells, cancer cells elevated ROS levels, thus altering the environment, making them more vulnerable to ROS-manipulation therapies. Disturbance in ROS levels changes cellular redox balance leading to oxidative stress, damage to mitochondria, and consequent apoptosis induction [49]. This may destroy cancer cells while sparing normal cells [46]. For instance, lanperisone, an identified compound, was able to act as a selective killer of Kras-mutant cancer cells that increased the steady-state levels of ROS [50]. As in our work, an article shows that apo-bLf treatment induces ROS production and depletion of cellular GSH on HeLa cells [48].

Caspases are aspartate-specific cysteine proteases that play essential roles in two main pathways that mediate apoptosis, the extrinsic/death and intrinsic-/mitochondria-dependent pathways [51–53]. Apoptosis or programmed cell death is a fundamental process for both health and disease that plays a vital role in carcinogenesis, immune system, embryonic development, maturation, and cytotoxic effector function [54]. Apoptosis promotion is one of the proposed mechanisms against cancer [35, 55].

The article "Bovine Lactoferrin Induces Cell Death in Human Prostate Cancer Cells" was published in 2022. Journal: Oxid Med Cell Longev.

We have shown evidence that bLf exhibited proapoptotic activities. Caspase 3/7 labeling was induced by apo-bLf and holo-bLf administration (Figure 5). CellEvent™ Caspase-3/7 assay used in this study is a substrate for activated caspases 3/7, so it is only fluorescent when caspases 3/7 are activated [56]. These results suggest that one of the mechanisms by which bLf engages their antitumor effects in prostate cancer is promoting apoptosis, thus corroborating with previous discoveries and cell viability experiments [35, 57].

Most of our results indicate that holo-bLf presented more antitumor effects when compared to apo-bLf. This was expected due to the conformation differences between apo- and holo-bLf [58]. The iron bond induces the structure to a more closed form; apo- has a more open and, consequently, more dynamic system than holo-. Thus, iron increases the stability of the protein since its structure is more closed and less susceptible to denaturation and proteolysis [4].

Thus, we can highlight the importance of using the holo- form of bLf in this work, since most papers use only the apo- form. Our results show that iron binding leads to an increase in the antitumor potential of this protein. New findings can expand the mechanism of action and protein expression involved in bLf effect. The results are relevant, as they will not only help research but will also contribute to a possible treatment for prostate cancer in the future. bLf has been shown to be very efficient against tumor cells *in vitro* studies, being an emerging biopharmaceutical [17, 21, 35–37]. Hence, some factors must be considered for its future use, as it may be a noninvasive and possibly preventive alternative for tumors. In addition, its low cost, mainly for public health systems, combined with its probable absence of side effects comparing to classic chemotherapy, makes bLf a promising candidate for antitumor.

Our results indicate that bLf may present antitumor activities by activating signaling pathways including, cell cycle arrest in the G_0_/G_1_ phase, apoptosis, and increase of ROS (Figure 6), thus corroborating with previous findings in the literature [35]. More studies on the apo- and holo-bLf mechanisms in cancer inhibition are needed.

## 5. Conclusions

In conclusion, the data presented in this work showed that treatments using bovine lactoferrin (apo- and holo-bLf forms) gave an antitumor effect in the prostate cancer cell line (DU-145). The holo-bLf form seems to be the substance with the highest potential for *in vivo* studies, thus offering a series of views on the use of these compounds in the prevention and treatment of prostate cancer, probably due to the iron binding. However, a more detailed investigation is needed to address better this issue and other cellular mechanisms activated by lactoferrin.

The article "Bovine Lactoferrin Induces Cell Death in Human Prostate Cancer Cells" was published in 2022. Journal: Oxid Med Cell Longev.

## Figures and Tables

**Figure 1:** Graphical scheme of the study approach.

**Figure 2:** bLf induces cell death in the DU-145 cell line. DU-145 cells were treated for 24 h and 48 h with 2, 4, 8, and 16 mg/mL of apo-bLf and holo-bLf. In the negative control, the culture medium was used. Values were plotted as percentages concerning the negative control, which represents 100% of viability. (a) MTT assay and apo-bLf treatment; (b) MTT assay and holo-bLf treatment; (c) trypan blue exclusion and apo-bLf treatment; (d) trypan blue exclusion and holo-bLf treatment. Graphs (a) and (b) represent two separate experiments with replicates. Graphs (c) and (d) represent three separate experiments. The experiment is expressed as mean ± SD. Significant differences between untreated and treated cells were compared using the one-way ANOVA test, with Bonferroni post hoc test (^∗^*p* < 0.05; ^∗∗^*p* < 0.01; ^∗∗∗^*p* < 0.001; ^∗∗∗∗^*p* < 0.0001).

**Figure 3:** bLf causes morphological changes in the DU-145 cell line. To verify the effects of bLf, selected images were taken using an EVOS microscope. (a) DU-145 cells were treated for 24 and 48 h with apo-bLf and holo-bLf at 8 and 16 mg/mL. (b) Zoom in of 8 mg/mL after 48 h treatment showing intracellular granules. The control cell received only a culture medium. The white bars represent a distance of 100 *μ*m. Arrowheads indicate stretched morphology.

**Figure 4:** bLf internalizes and causes DU-145 cell damage. DU-145 cells were incubated with apo- and holo-bLf labeled with FITC for 24 h at 8 and 16 mg/mL concentrations. The images were obtained using fluorescence confocal microscopy (LSM 510 META Confocal Laser Scanning Microscope) and EC Plan-Neofluar 40x/1.30 Oil DIC M27 (Zeiss Inc.) objective lens. The white bars represent a distance of 40 *μ*m.

**Figure 5:** DU-145 cell treatment with apo- and holo-bLf induces oxidative stress and activates caspases 3/7. Cells were treated with 2, 4, 8, and 16 mg/mL of apo- and holo-bLf for 24 and 48 h and analyzed in high-throughput system Operetta. (a) Oxidative stress with apo-bLf treatment through dihydroethidium- (DHE-) labeled cell. (b) Oxidative stress with holo-bLf treatment through dihydroethidium- (DHE-) labeled cell. (c) Caspases 3/7 activation with apo-bLf treatment through CellEvent Caspase 3/7 Green Detection Reagent. (d) Caspases 3/7 activation with holo-bLf treatment through CellEvent Caspase 3/7 Green Detection Reagent. These graphics represent one distinct experiment with replicates. The experiment is expressed as mean ± SD. Significant differences between untreated and treated cells were compared by the one-way ANOVA test, with Bonferroni post hoc test (^∗^*p* < 0.05; ^∗∗^*p* < 0.01; ^∗∗∗^*p* < 0.001; ^∗∗∗∗^*p* < 0.0001).

The article "Bovine Lactoferrin Induces Cell Death in Human Prostate Cancer Cells" was published in 2022. Journal: Oxid Med Cell Longev.

**Figure 6:** General scheme of the bLf effects on DU-145 cells. Diagram indicates internalization of bLf (apo- and holo-), increased oxidative stress, induction of morphological changes, apoptosis, and cell cycle arrest in the G_0_/G_1_ phase.

**Table 1:** bLf modulates cell cycle of DU-145 cell line. The table below shows the percentage of cells in each cell cycle phase determined by flow cytometry. This table represents three different experiments expressed as mean ± SD. The one-way ANOVA test compared significant differences between untreated and treated cells with the Bonferroni post hoc test.

	24 h treatment			48 h treatment		
	G_0_/G_1_ (%)	S (%)	G_2_/M (%)	G_0_/G_1_ (%)	S (%)	G_2_/M (%)
Control	44.1 ± 3.6	27.5 ± 5.4	13.9 ± 0.9	46 ± 6.9	22.7 ± 8.8	14.4 ± 3.6
Apo-bLf 2 mg/mL	45.4 ± 2.8	22.9 ± 6.8	13.3 ± 2.5	54.2 ± 7.4	17 ± 7.1	12.4 ± 3.7
Apo-bLf 4 mg/mL	41.1 ± 2.2	26.3 ± 4.5	13.8 ± 1.1	51.6 ± 5.4	18.9 ± 5.2	13.5 ± 3.6
Apo-bLf 8 mg/mL	42.4 ± 5.4	23.3 ± 3.9	14.4 ± 1.3	53.4 ± 3.4	18 ± 7.7	14.3 ± 4.9
Apo-bLf 16 mg/mL	53.7 ± 1.4	20.5 ± 1.2	13.3 ± 2.4	50.5 ± 3.7	18.8 ± 4.9	12.8 ± 6.1
Holo-bLf 2 mg/mL	46.9 ± 9.5	24.4 ± 7.3	15.3 ± 2.5	56.2 ± 4.7	18.6 ± 9.8	15.1 ± 2.3
Holo-bLf 4 mg/mL	47.1 ± 6.6	22.3 ± 5.3	16.4 ± 3.5	57.2 ± 3.8	19.3 ± 9.1	15.4 ± 2.1
Holo-bLf 8 mg/mL	51.4 ± 4.3	21.3 ± 1.4	13.9 ± 1.9	63.5 ± 4.5	18 ± 6.7	12.4 ± 1.6
Holo-bLf 16 mg/mL	67.0^a^ ± 11.3	14 ± 4.7	11.3 ± 4.1	75.4^b^ ± 9.9	11.3 ± 3.8	10.8 ± 4.2

^∗^Different letters indicate statistical difference compared to control (^a^*p* < 0.05; ^b^*p* < 0.01).

## Data Availability

The data used to support the findings in this paper are available from the corresponding author upon request.
